# Efficacy of Fluticasone and Salmeterol Dry Powder in Treating Patients with Bronchial Asthma and Its Effect on Inflammatory Factors and Pulmonary Function

This article has been retracted.

**DOI:** 10.1155/2022/8555417

**Published:** 2022-08-11

**Authors:** Xiaodan Zhang, Min Liu, Yuhong Mao

**Affiliations:** ^1^Department of Basic Disciplines, Jiangxi Health Vocational College, Nanchang, Jiangxi 330052, China; ^2^Department of Respiratory and Critical Care Medicine, The Affiliated Nanhua Hospital, Hengyang Medical College, University of South China, Hengyang, Hunan 421001, China

## Abstract

**Objective:**

To evaluate the efficacy of fluticasone and salmeterol dry powder in treating patients with bronchial asthma and its effects on inflammatory factors and pulmonary function.

**Methods:**

One hundred patients with bronchial asthma, admitted to our hospital between April 2019 and June 2020, were enrolled and assigned into two groups using the random number table method. The observation group (*n* = 50) received budesonide powder, and the experimental group received fluticasone and salmeterol dry powder. The two groups were compared with regard to clinical efficacy, inflammatory factors, pulmonary function, and adverse reactions.

**Results:**

In the experimental group, the total effective rate of treatment was significantly higher than that in the observation group (*P* < 0.05); after treatment, the levels of inflammatory factors in the experimental group were lower than those in the observation group (*P* < 0.05); after treatment, lung function in the experimental group was significantly higher than that in the observation group (*P* < 0.05); the incidence of adverse reactions in the experimental group was significantly lower than that in the observation group (*P* < 0.05).

**Conclusion:**

Salmeterol and fluticasone powder has shown impressive clinical benefits in the treatment of bronchial asthma patients. It might be a viable approach to reduce inflammatory factors and improve pulmonary function. Moreover, its good clinical safety profile makes it a promising treatment that ought to be promoted and used widely.

## 1. Introduction

Clinical respiratory medicine considers bronchial asthma to be one of the most common pathological forms, mostly caused by the heterogeneity of the body's cells [1]. A cascade of factors is accountable including physiology and environment [2]. The main symptoms of bronchial asthma are shortness of breath, sudden wheezing, cough, and chest discomfort [3]. The disease is more common in individuals with allergic constitutions and individuals with low resistance [4].

For the treatment of bronchial asthma, salmeterol and fluticasone powder and budesonide powder are both commonly used drugs. Although both can significantly mitigate the symptoms of patients, budesonide powder is too irritating, which may increase the risk of adverse reactions in patients [5]. In recent years, salmeterol and fluticasone powder has emerged as a mainstay for bronchial asthma, and the drug is composed of fluticasone propionate and salmeterol [6]. Since the former aims to improve lung function, the latter targets to improve patients' overall health, these two treatments complement one another [7]. To this end, we hypothesized in this study that salmeterol and fluticasone powder in the treatment of patients with bronchial asthma yields a promising result in inflammatory factors and lung function.

## 2. Data and Methods

### 2.1. Baseline Data

The study population was 100 patients with bronchial asthma admitted to our hospital from April 2019 to June 2020, who were equally divided into the observation group (*n* = 50) and the experimental group (*n* = 50) using the random number table method. All patients themselves and their families were informed of the study and signed consent forms, and the study was approved by the ethics committee (Approval No. 20192524).

### 2.2. Inclusion and Exclusion Criteria

#### 2.2.1. Inclusion Criteria

1. Bronchial asthma was diagnosed in all patients by clinical examination [8]
2. Patients without other serious heart diseases
3. The patients were informed about the study and voluntarily participated in it
4. The patient has not used glucocorticoids 30 days before treatment, *β*2-receptor agonists within 7 days, or other asthma drugs except albuterol aerosol within 15 days
5. Patients with no abnormal liver and kidney function, severe gastrointestinal diseases, blood diseases, and malignant tumors

#### 2.2.2. Exclusion Criteria

1. Patients with other serious medical conditions
2. Patients with poor compliance who are unwilling to participate in the study
3. Patients who are unconscious or have other mental illnesses
4. Patients who have had serious adverse reactions to the drugs used in the experiment
5. Pregnant and lactating women

### 2.3. Methods

In both groups, fluid rehydration, anti-infection, spasmolysis, and aminophylline were administered as symptomatic treatment. In the observation group, budesonide powder (Xinyi Baluda Pharmaceutical Co., Ltd., National Drug Approval H20080316, specification: 0.2 mg) was administered twice daily at a dose ranging from 0.4 to 1.2 mg. The experimental group was given daily doses of salmeterol and fluticasone powder twice (Glaxo Operations UK Limited, National Drug Approval H20090242, Specification: 55 *μ*g), 55 *μ*g each time. Both groups underwent treatment for six months.

### 2.4. Observational Indicators

#### 2.4.1. Clinical Efficacy: Markedly Effective

A marked improvement in the patient's asthma attack was noted, and his breathing was smooth. Effective: the asthma attack of the patient has been relieved; there are, however, occasional instances of difficulty breathing. Ineffective: the condition has failed to improve or worsen.

#### 2.4.2. Levels of Inflammatory Factors

The level of inflammatory factors (tumor necrosis factor (TNF-*α*), interleukin-4 (IL-4), and IL-8) in patient serum was assessed by enzyme-linked immunosorbent assay (Thermo Fisher) after routine centrifugation of 5 mL of fasting venous blood collected before and after treatment.

#### 2.4.3. Pulmonary Function

The pulmonary function tests were performed using a spirometer (Jaeger, Germany) including 1s forced expiratory volume (FEV1), forced vital capacity (FVC), and peak expiratory flow (PEF).

#### 2.4.4. Adverse Reactions

The potential adverse reactions were defined as follows: patient's health has not improved or has worsened, such as severe discomfort, rash, and oropharyngeal irritation.

### 2.5. Statistical Analysis

SPSS20.0 was used for the analysis of the data. Measurement data were expressed as $\left(\bar{x}\pm s\right)$ and the independent sample *t*-tests were used for the comparison. Enumeration data were expressed as the number of cases (%) and the *x*^2^ test was utilized for the comparison. Significance was determined with *P* values less than 0.05. The mapping software used was GraphPad Prism 8.

## 3. Results

### 3.1. Baseline Data

The observation group consisted of 31 males and 19 females; ages ranged from 24 to 59 years, with an average age of 41.28 ± 3.45 years; the disease course ranged from 1 to 13 years, with an average duration of 7.14 ± 1.28 years. There were 33 males and 17 females in the experimental group; their ages ranged from 23 to 60 years, with an average age of 41.34 ± 3.52 years. There was no significant difference between the two groups of patients in terms of the general data (*P* > 0.05), as shown in Table 1.

### 3.2. Comparison of Clinical Efficacy

Compared to the control group, the total effectiveness rate in the experimental group was significantly higher (*P* < 0.05), as shown in Table 2.

### 3.3. Comparison of Inflammatory Factors

Before treatment, there was no substantial difference in inflammatory factors between the experimental and observation groups (*P* > 0.05); after treatment, inflammatory factors in the experimental group were lower than those in the observation group (*P* > 0.05) (Figure 1).

### 3.4. Comparison of Pulmonary Functions

Significant differences did not exist between the two groups in terms of pulmonary function indexes before treatment (*P* > 0.05); the pulmonary function indexes of the experimental group were higher than those of the observation group after treatment (*P* < 0.05), as shown in Figure 2.

### 3.5. Comparison of Adverse Reactions

In the experimental group, adverse reactions were significantly less frequent than those in the observation group (*P* < 0.05) (Table 3).

## 4. Discussion

The incidence of bronchial asthma in China has been on the rise as a result of the ever-worsening environmental pollution. The contributors to bronchial asthma include inflammatory cytokines and chronic inflammatory factors [9]. Moreover, genetics and the environment are two essential factors in the pathogenesis of asthma patients, among which genetics only determines the allergic constitution of patients, that is, prone to asthma, and environmental factors play a crucial role [10]. Early symptoms of bronchial asthma include coughing, chest tightness, and dyspnea, and dry cough and white foamy sputum may occur in severe cases [11]. The disease has high clinical morbidity and is relapsing, which significantly affects the daily lives of patients [12]. Asthma cannot be cured, and drug treatment is generally used, and it is divided into control drugs and relievers [13]. Controller medications require long-term use of daily medications that maintain clinical control of asthma primarily through anti-inflammatory effects, including inhaled corticosteroids, systemic corticosteroids, long-acting beta 2 agonists, anti-IgE monoclonal antibodies, and other asthma-lowering drugs [14]. Reliever medications, also known as rescue medications, relieve asthma symptoms by rapidly relieving bronchospasm, including fast-acting inhaled and short-acting oral beta 2 agonists, systemic corticosteroids, inhaled anticholinergics, and short-acting theophylline [15].

Currently, hormonal anti-inflammatory drugs are used to treat patients with bronchial asthma in clinical settings. In treating patients with bronchial asthma, budesonide powder is a commonly used medication. Budesonide is a cortical anti-inflammatory drug that can effectively alleviate inflammatory responses in patients' bodies. Nonetheless, budesonide has a high affinity for glucocorticoid receptors, which can significantly reduce the amount of budesonide entering the patient's body [16]. According to the research of Wang (2020), budesonide powder can effectively treat allergic-induced inflammatory diseases and effectively control inflammatory factors, but the outcome remains insufficiently ideal for patients who suffer from recurrent bronchial asthma. Salmeterol and fluticasone powder is a new common drug that has been used in the treatment of bronchial asthma in recent years [17, 18]. It has been demonstrated that salmeterol (*β*2 receptor agonist) has a significant dilating effect on the bronchi of patients [19]. The release of pulmonary mast cell mediators such as triene and histamine is the basis for improvement and remission of the patient's disease condition, while fluticasone propionate is one of the glucocorticoids with strong water- and fat-soluble properties [20]. It can have an anti-inflammatory effect on the patient's body and clinical studies have confirmed that it does not cause any adverse effects [21].

The results of the present study demonstrated that the clinical efficacy of the experimental group was significantly higher than that of the observation group; the adverse reactions of the experimental group were significantly less than those of the observation group. Moreover, salmeterol fluticasone has a significant clinical effect and has a high safety profile in the treatment of patients with bronchial asthma. The possible explanation is the fact that salmeterol and fluticasone powder has a fast onset and long drug effect on patients, and it can directly act on them. Taking the drug through the patient's smooth muscle allows the patient's body membrane to absorb the drug completely, and the salmeterol in the drug can cause the bronchi to relax for a long period of time, helping the patient ease bronchospasm, thus improving their symptoms of disease [22]. Compared with the budesonide powder, the salmeterol and fluticasone powder has less irritation to the patient's body, and its dose is simpler to control, so its clinical treatment safety is higher. As previously noted, the level of inflammatory factors in the body is closely correlated with the recurrence of bronchial asthma in clinical studies. Ewing et al. have demonstrated that reducing the level of inflammatory factors in patients with bronchial asthma can effectively prevent recurrence [23]. Gans and Gavrilova found that improving lung function indicators in patients with bronchial asthma can significantly enhance the effect of treatment and improve their quality of life [24]. As part of this study, we compared the levels of inflammatory factors and pulmonary function between the two groups of patients and found that the inflammatory factors in the experimental group were significantly lower than those in the observation group after treatment. Presumably, the main component of salmeterol and fluticasone propionate are salmeterol and fluticasone propionate. In contrast, the latter is a new type of long-acting *β*2 receptor agonist that has the ability to effectively stimulate the biological activity of the adenosine activating enzyme in the body's cells, resulting in much faster conversion of adenosine triphosphate within the human body. This can result in a decrease in the body's cyclic adenine phosphate concentration, reducing bronchospasm, and improving lung function. Promisingly, salmeterol's effect lasts for a long time, ensuring that the patient enjoys persistent effectiveness of the drug throughout the night [25]. Fluticasone propionate is a glucocorticoid, which can bind to the glucocorticoid receptor in the local inflammatory response area of the patient's body, so that the patient's body is able to produce steroids to inhibit epithelial cell growth and the expression of inflammatory factors, thereby providing anti-inflammatory action. Salmeterol is capable of significantly improving the sensitivity of the patient's body to glucocorticoids, thereby enhancing the efficacy of fluticasone propionate. Additionally, it can reduce the levels of inflammatory factors in the patient's body [26].

According to traditional Chinese medicine (TCM), asthma is a disease with the main symptoms of phlegm in the throat, dyspnea, and even the inability to lie down due to wheezing [27]. TCM treatment of asthma requires staging and syndrome differentiation. In essence, responding to the different stages of patients, different treatment measures should be taken to effectively relieve symptoms. For instance, symptomatic treatment can be taken in acute attack, while in the remission stage, root-consolidating treatment can be adopted [28, 29]. TCM treatment of asthma mainly includes dispelling wind and dissipating heat, clearing heat and dispersing the lungs, and resolving phlegm and relieving asthma. [30]. Asthma attack is mostly caused by exogenous cold, interaction of internal and external pathogens, and stagnation of phlegm and qi, and it is generally treated with Xiaoqinglong soup or Ma Hengshi Gan soup [31]. In the remission phase of asthma, the spleen should be tonified, the kidney should be benefited, and phlegm should be dispelled to calm asthma, and Sheng Wei San and Ginseng and Bai Zhu San can be used [32].

However, we need further research to more accurately determine the role of combination therapy, especially the dose-related issues, to examine the potential systemic side effects. Despite the current recommendations that are primarily resulted from clinical trials, the potential benefits of combination therapy may lead to changes in these recommendations. We are firmly convinced that understanding the mechanisms of the interactions may provide insights into the development of more effective therapies.

## 5. Conclusion

In conclusion, the combination of salmeterol and fluticasone powder yields a pronounced efficiency in the treatment of patients with bronchial asthma. It mitigates the inflammatory reactions and improves pulmonary function, which warrants a wide promotion.

## Figures and Tables

**Figure 1:** Comparison of inflammatory factors $\;\left(\bar{x}\pm s\right)$.

**Figure 2:** Comparison of pulmonary functions $\;\left(\bar{x}\pm s\right)$.

**Table 1:** Comparison of general data [*n*(%)].

	Observation group (*n* = 50)	Experimental group (*n* = 50)	*t*/*x*^2^	*P*
Gender			0.174	0.677
Male	31	33		
Female	19	17		
Age (years)	24–59	23–60		
Average age (years)	41.28 ± 3.45	41.34 ± 3.52	−0.086	0.932
Disease course (years)	1–13	1–14		
Average course of disease (years)	7.14 ± 1.28	7.29 ± 1.36	−0.568	0.571

**Table 2:** Comparison of clinical efficacy [*n*(%)].

	Observation group (*n* = 50)	Experimental group (*n* = 50)	*x * ^2^	*P*
Markedly effective	24	38		
Effective	15	11		
Ineffective	11	1		
Overall response rate (%)	39 (78%)	49 (98%)	9.47	0.002

**Table 3:** Comparison of adverse reactions [*n*(%)].

	Observation group (*n* = 50)	Experimental group (*n* = 50)	*x * ^2^	*P*
Hoarse voice	3	1		
Skin rash	1	0		
Oropharyngeal irritation	5	1		
Overall rate (%)	9 (18%)	2 (4%)	5.005	0.025

## Data Availability

All data generated or analysed during this study are included in this published article.
